# Bone Marrow Plasma Cytokine Signature Profiles in Severe Aplastic Anemia

This article has been retracted.

**DOI:** 10.1155/2020/8789275

**Published:** 2020-02-18

**Authors:** Bingnan Liu, Yuanyuan Shao, Zixuan Liu, Chunyan Liu, Tian Zhang, Rong Fu

**Affiliations:** Department of Hematology, Tianjin Medical University General Hospital, 154 Anshan Street, Heping District, Tianjin 300052, China

## Abstract

**Objective:**

We studied bone marrow plasma (BMP) cytokines in severe aplastic anemia (SAA) patients and healthy volunteers to investigate differences in the cytokine profiles between them and propose a cytokine signature of SAA.

**Methods:**

A Bio-Plex suspension array system was used to measure 27 analytes in BMP samples from 47 SAA patients and 30 healthy donors.

**Results:**

Compared to healthy people, SAA patients had higher levels of tumor necrosis factor *α* (TNF-*α* (TNF-*γ* (IFN-*γ* (IFN-*β* (MIP-1*β* (MIP-1*α* (TNF-*α* (TNF-*β* (MIP-1*β* (MIP-1*β* (MIP-1*γ* (IFN-*α* (TNF-

**Conclusions:**

The current study demonstrated distinct cytokine profiles among untreated SAA patients, recovering SAA (RSAA) patients, and healthy people. The cytokines of RSAA patients showed similar characteristics to those of untreated SAA patients and healthy people, respectively, which may reflect that the immune status of RSAA patients is in different stages of recovery after IST; thus, it may provide an important tool in diagnosing and evaluating or predicting curative effects in clinics.

## 1. Introduction

Severe aplastic anemia (SAA) is a severe disease characterized by bone marrow failure and a high fatality rate. Bone marrow failure in SAA is usually caused by an immunologic mechanism, and immunosuppressive therapy (IST) is effective in most SAA patients [1, 2]. Cytokines and chemokines play a key role in immune cell activation in the pathogenesis of SAA. Cytokines and chemokines are low-molecular-weight proteins that are secreted by immunocytes, activate other immune cells, and mediate inflammatory responses. Previous studies have shown that CD8^+^T cells are aberrantly activated in SAA as myeloid dendritic cells (mDCs) and helper Th1 cells [2, 3]. Meanwhile, IFN-*γ*, TNF-*α*, and IL-2 levels have been shown to significantly increase in SAA [4, 5]. Although the immune pathogenesis of SAA has been widely studied, very little is known about the alternations of cytokines and chemokines in the bone marrow.

In the past, measurements of cytokines have been limited to two or three in SAA [6]. Due to the large number of proteins involved in the immune reaction, the detection of a single cytokine is not enough to evaluate the change in disease. Based on this, we conducted a comprehensive testing of 27 cytokines and chemokines in the bone marrow plasma (BMP) of healthy volunteers, untreated SAA patients, and recovering SAA (RSAA) patients. We describe differences in the cytokine profiles between these groups and propose a cytokine signature that might help in exploring the pathogenesis of SAA.

## 2. Patients and Methods

### 2.1. Patients

Forty-seven patient samples and thirty healthy control (HC) samples were measured in the present study. This cohort of patients included 28 SAA patients who were previously untreated and 19 RSAA patients. SAA was diagnosed according to the criteria of the International Aplastic Anemia Study Group [7]. Participants who had paroxysmal nocturnal hemoglobinuria, myelodysplastic syndrome, tumors, infections, or congenital diseases were excluded. Patients with SAA were diagnosed in our department from March 2018 to August 2019. In six of the untreated SAA patients, serial analyses were performed before and three and six months after rabbit anti-human thymocyte immunoglobulin (rATG) and cyclosporine (CsA) treatment. RSAA patients were defined as SAA patients having experienced substantial improvement after therapy with rATG (Fresenius, Germany) and a decreasing dose of CsA [8]; all of these patients became completely transfusion-independent. The clinical characteristics of the patients are listed in Table 1. Healthy volunteers were recruited from the staff of our laboratory and health examination center. The 77 samples included samples from 36 males and 41 females, with ages ranging from 11 to 78 years and a median age of 36 years. The study procedures and informed written consent were approved by the Ethics Committee of Tianjin Medical University.

### 2.2. Cytokine and Chemokine Measurement

Plasma samples were obtained by centrifugation of heparinized bone marrow and stored at −80°C until examination. We analyzed 27 cytokines and chemokines in the BMP of the samples by applying Luminex-based multiplex bead technology. The Bio-Plex Pro Human Cytokine group I Panel 27-Plex was applied out as follows: IL-1*β*, IL-1ra, IL-2, IL-4, IL-5, IL-6, IL-7, IL-8 (CXCL-8), IL-9, IL-10, IL-12p70, IL-13, IL-15, IL-17, basic fibroblast growth factor (FGF-*β*), eotaxin (CCL-11), granulocyte colony-stimulating factor (G-CSF), granulocyte-macrophage colony-stimulating factor (GM-CSF), IFN-*γ*, IFN inducible protein-10 (IP-10; CXCL-10), MCP-1 (CCL-2), macrophage inflammatory protein 1*α* (MIP-1*α*; CCL-3), MIP-1*β* (CCL-4), platelet-derived growth factor-BB (PDGF-BB), RANTES (CCL-5), TNF-*α*, and vascular endothelial growth factor (VEGF; Bio-Rad Laboratories, Inc., Made in the USA). All Bio-Plex assays were conducted according to the manufacturer's instructions. The median fluorescence intensities (MFIs) of analytes were analyzed on a Luminex-100 instrument (Luminex, Bio-Rad) using Bio-Plex Manager software version 6.0 (Bio-Rad, USA). Each analyte was tested in duplicate, and the average value was recorded as the measured concentration. The acquired data was processed by applying Data Pro Manager 1.02 (Bio-Rad, USA) and Prism Software version 6.0.

### 2.3. Statistical Analysis

When the normality of the distribution was proven using a Kolmogorov-Smirnov test, an independent *t*-test was used to compare the means of the analyte concentrations; otherwise, a nonparametric test was applied. For the nonnormal distribution data, a Mann–Whitney *U* test was used to compare two groups of continuous variables and a Kruskal–Wallis one-way ANOVA was used to compare three groups. In drawing a cluster heat map, a log transformation was applied to the data to correct for nonnormal distribution. A Spearman's rank correlation test was used to test for correlated data; when significant results were found, the correlation coefficient (*r*) was reported. Quantitative data was expressed in the form of means ± SDs and medians, and significance was considered when *p* < 0.05. SPSS 19.0 software (IBM, USA) was used for statistical analyses.

## 3. Results

### 3.1. BMP Cytokine Concentration in SAA Patients and Healthy Controls

Cytokine Bio-Plex assays were conducted to measure the BMP cytokine concentrations in SAA patients and HCs. The median cytokine concentrations of the SAA patients, RSAA patients, and HCs are shown in Figure 1; the mean, standard deviation (SD) of the mean, and median values are presented in Table 2. As shown in Figure 1, higher levels of TNF-*α*, IFN-*γ*, G-CSF, IL-2, and MCP-1 (Figures 1(a)–1(f)) and lower levels of IL-1ra, PDGF-BB, IL-9, RANTES, and MIP-1*β* (Figures 1(g)–1(n)) were present in SAA patients compared to HCs. Additionally, levels of IL-1ra, eotaxin, and MIP-1*α* were significantly higher in RSAA patients than those in HCs (Figures 1(g), 1(i), and 1(m)). The median concentration of IFN-*γ* in untreated SAA patients was 3.56 ng/ml, which was higher than that found in recovery patients (1.69 ng/ml) and normal controls (1.51 ng/ml; *p* < 0.001; Figure 1(b)). The median concentration of RANTES in untreated SAA patients was 203.775 ng/ml, which was significantly lower than that found in RSAA patients (1222.56 ng/ml) and HCs (1903.03 ng/ml; *p* < 0.001; Figure 1(l)). The median concentrations of IL-1ra in SAA patients, RSAA patients, and HCs were 39.955 ng/ml, 120.72 ng/ml, and 54.55 ng/ml, respectively; the level of IL-1ra found in recovery patients was higher than that found in untreated patients (*p*=0.002; Figure 1(g)). Levels of IL-5, IL-6, IL-10, IL-12p70, IL-13, IL-15, GM-CSF, and VEGF were undetectable. Additionally, there were no significant differences in IL-1*β*, IL-4, IL-7, IL-8, IL-17, FGF-*β*, and IP-10 levels between the SAA patients and the HCs.

Compared to the RSAA patients and HCs, the SAA patients had higher levels of Type I lymphocyte factor secreted by T-helper cell 1 (Th1). IL-2, IFN-*γ*, and TNF-*α* levels were the highest among the SAA patients, with no differences between those of the RSAA patients and those of the HCs, and the IL-7 levels showed an increasing trend (*p*=0.087) in the SAA patients (Figures 1(a), 1(b), and 1(d)). In contrast, we found an increasing trend of IL-4 levels (representative of Th2 cytokine) in the RSAA group, although this trend was not statistically significant (*p*=0.098). The Th1/Th2 cytokine ratio of IFN-*γ* to IL-4 was significantly higher in the SAA group than that in the other groups (Figure 1(e)). Furthermore, MCP-1 (a Th2 cytokine) was the highest in the SAA patients (*p* < 0.001) but more elevated in the RSAA patients (*p*=0.020) than in the HCs (Figure 1(f)). Among the cytokines that were the lowest in the SAA patients, IL-9 and PDGF-BB (Figures 1(j) and 1(k)) were also lower in the RSAA patients but MIP-1*β* and RANTES (Figures 1(l) and 1(n)) appeared to be higher in the RSAA patients and there were no statistic differences between RSAA and HC.

To classify cytokine patterns among the individuals, we performed a two-way hierarchical cluster analysis on log-transformed data from the SAA patients, RSAA patients, and HCs using OriginPro 2018 (Figure 2). The dendrogram above Figure 2 was categorized into three clusters, conforming to the corresponding groups for the majority of samples, which indicated that the SAA patients, RSAA patients, and HCs showed different cytokine patterns. Meanwhile, the overlaps of the three clusters implied that the cytokine pattern of some RSAA patients had not been recovered, while others had returned to normal. The dendrogram to the left of Figure 2 displayed the proximity between the different cytokines. The cluster heat map showed four groups of cytokines: (1) IL-7, TNF-*α*, MCP-1, IFN-*γ*, IL-2, and G-CSF; (2) IP-10, RANTES, PDGF-bb, and IL-9; (3) MIP-1*β*, MIP-1*α*, IL-8, and IL-1ra; and (4) eotaxin, IL-17, IL-4, FGF-*β*, and IL-1*β*. Cytokines in each of these groups may play proximate roles and/or share the same origin.

### 3.2. Correlation of BMP Cytokine Concentrations with Clinical Parameters

A Spearman correlation analysis was performed to investigate the correlation of BMP cytokines with blood cell levels in SAA and RSAA patients (Table 3). MIP-1*α* and RANTES levels correlated significantly with major blood cell types including absolute neutrophil count (*r* = 0.481, *p*=0.001; *r* = 0.291, *p*=0.047), hemoglobin (*r* = 0.389, *p*=0.007; *r* = 0.414, *p*=0.004), platelet count (*r* = 0.360, *p*=0.013; *r* = 0.442, *p*=0.002), proportion of reticulocytes (*r* = 0.510, *p* < 0.001; *r* = 0.451, *p*=0.001), and absolute reticulocyte count (*r* = 0.595, *p* < 0.001; *r* = 0.505, *p* < 0.001). IL-1ra, eotaxin, G-CSF, and MIP-1*β* also significantly correlated with major blood cell types, except for hemoglobin, including absolute neutrophil count (*r* = 0.481, *p*=0.001; *r* = 0.291, *p*=0.047), platelet count (*r* = 0.360, *p*=0.013; *r* = 0.442, *p*=0.002), proportion of reticulocytes (*r* = 0.510, *p* < 0.001; *r* = 0.451, *p*=0.001), and absolute reticulocyte count (*r* = 0.595, *p* < 0.001; *r* = 0.505, *p* < 0.001). Notably, IL-2, G-CSF, IFN-*γ*, and TNF-*α* negatively correlated with the aforementioned parameters, whereas the other cytokines correlated positively with these parameters. Among these cytokines, IFN-*γ* correlated more strongly with absolute neutrophil count (*r* = −0.307, *p* < 0.001) than did hemoglobin, platelet count, proportion of reticulocytes, or absolute reticulocyte count; TNF-*α* correlated more strongly with platelet count (*r* = −0.320, *p*=0.028) than did other cell types; and IL-2 correlated more strongly with absolute neutrophil count (*r* = -0.393, *p*=0.006), platelet count (*r* = −0.355, *p*=0.014), and absolute reticulocyte count (*r* = −0.319, *p*=0.029) than did other cell types.

### 3.3. BMP Cytokine Concentration and Age/Gender

There were no significant differences in the levels of IL-1*β*, IL-4, IL-7, IL-8, IL-17, FGF-*β*, and IP-10 between the patients and the HCs. To explore what factors might have caused these cytokine levels to differ between individuals, we analyzed the correlations of age and gender with cytokine concentrations in all samples. We performed a Spearman test to explore the correlation of cytokine concentration with age. The results of this test showed that the levels of three cytokines were significantly and positively correlated with age: IL-8 (*r* = 0.225, *p*=0.049), IP-10 (*r* = 0.218, *p*=0.049), and FGF-*β* (*r* = 0.278, *p*=0.014; Figures 3(a)–3(c)).

We conducted a Mann–Whitney test to evaluate the differences in cytokine concentrations between gender groups in all samples (36 males, 41 females). Only one BMP cytokine concentration was different between men and women: the median concentration of IL-17 was higher in men than in women (6.79 pg/mL versus 4.01 pg/mL; *p*=0.048; Figure 3(d)).

### 3.4. BMP Cytokine Concentrations in SAA Patients before and after IST

In order to determine whether there were any changes in the cytokine levels of SAA patients after receiving IST, we detected the cytokine levels of six patients before and three and six months after receiving ATG + CsA treatment (Figure 4). Statistically significant increases in eotaxin, IL-1ra, and MCP-1 had occurred by three months after IST. MIP-1*β* and RANTES levels had increased by six months after IST. IFN-*γ* and G-CSF concentrations, which were the highest in the untreated SAA patients, had decreased by three months after IST. Decreases in IL-2, IL-7, and TNF-*α* were observed by six months after IST.

## 4. Discussion

In the present study, increased levels of Type I lymphocyte factors IFN-*γ*, IL-2, and TNF-*α* were observed in the BMP of untreated SAA patients; these levels decreased after IST. These results are consistent with the theory of SAA immune pathogenesis, which suggests that SAA is an autoimmune disease that results from overactivation of the immune system, especially T lymphocytes [1, 2]. Cytokines are also excessively secreted by T cells, indicating that the pathogenesis of SAA is associated with the Th1 cell response [4, 5]. In addition, the immune pathogenesis of SAA also includes imbalance dendritic cell subsets (elevated mDC), enhanced dendritic cell function, insufficiency of Treg cells, and decreased proportion but enhanced function of NK cells [3, 10]. However, the IL-12 and GM-CSF involved in these immune processes were undetectable in all samples. A significant increase in G-CSF was also observed in SAA patients. The elevated concentrations of G-CSF in SAA patients may reflect a physiological negative feedback mechanism; this conclusion is consistent with those of previous studies [11]. Because Th2 cytokines showed an increasing trend in SAA and RSAA patients without statistically significant difference between the groups, we compared the Th1/Th2 cytokine ratio of IFN-*γ* to IL-4 between three groups, and the result of this comparison indicated that the SAA group had a significantly higher ratio of IFN-*γ* to IL-4 than did the RSAA and HC groups. Most Th2 cytokines, including IL-6, IL-5, IL-13, and IL-10, were undetectable in the present study. Monocyte chemoattractant protein-1 (CCL-2/MCP-1) is an important chemokine that regulates the migration and infiltration of macrophages/monocytes [12]. Although levels of MCP-1 (a Th2 cytokine) were significantly higher in SAA and RSAA patients than those in HCs, serial measurements before and after IST showed that MCP-1 concentrations increased after three months, indicating that both Th1 and Th2 cytokines increased in SAA patients but Th1 predominated.

Besides Th1/2 cytokines, there were a few studies about other cytokines in SAA. Our analysis revealed that the levels of PDGF-BB and IL-9 were significantly lower in both SAA and RSAA patients than those in HCs. Concentrations of RANTES and MIP-1*β* were significantly lower in SAA patients than those in RSAA patients and HCs; these concentrations also increased after IST.

Results concerning the functions of PDGF-BB in SAA were consistent with the results of studies concerning other diseases such as severe sepsis [13]. PDGF-BB is a cytokine that was found in this study to inhibit the activation of immunocytes and the production of cytokines *in vivo* and *in vitro*. PDGF-BB concentration was negatively correlated with proinflammatory cytokine (TNF-*α*, IL-1*β*, and IL-8) and chemokine (CXCL-1 and MCP-1) concentrations.

IL-9 levels have been reported to be higher in some tumors, such as multiple myeloma tumors, than those in the controls; however, IL-9 has complicated dual functions in different tumors [14]. IL-9 provokes an inflammatory environment promoting CD8^+^ cytotoxic T lymphocyte activation in tumor tissues of melanoma models but is also involved in tumor immune tolerance in breast cancer [15]. Therefore, IL-9 has been proven to trigger physiological immune responses in terms of both innate and adaptive immunity but is not limited to any one function. In SAA, lower levels of IL-9 may indicate that the immune process is different from the way that in the tumor.

RANTES and MIP-1*β* were included in the CC family of chemokines. One study suggested that MIP-1*α*, MIP-1*β*, and RANTES are cosecreted to a large extent with IFN-*γ* by activated CD4^+^ Th1, CD8^+^T, and NK cells *in vitro* and in a model of murine listeriosis [16]. RANTES, MIP-1*α*, IFN-*γ*, and MIP-1*β* were considered together as a *functional unit* driving the Th1 immune response to certain pathogens by NK and CD8^+^ T cells *in vivo* [16]. However, our data showed the opposite result in that RANTES and MIP-1*β* were significantly lower in SAA patients than those in RSAA patients and HCs. Besides the differences between *in vitro* and *in vivo* and between human and murine studies, it may be indicated that the antigens provoking immune progress were not a specific pathogen in SAA. In addition, a study with similar results to ours showed that elevated pre-antiretroviral-therapy MIP-1*β* levels identified long-term immunological nonresponse in HIV-infected patients, indicating that MIP-1*β* might be of use in the early identification of long-term immunological nonresponse [17]. MIP-1*α* levels were lower in SAA patients, although the RSAA group had significantly higher MIP-1*α* levels. This result was consistent with the results of a study on the expression of hematopoietic regulatory molecules in bone marrow mesenchymal stem cells induced by lipopolysaccharides in aplastic anemia patients [18]. Another study revealed that the endogenous MIP-1*α* promoter contains two consensus Runt-domain transcription factor (RUNX) sites in humans that are able to bind to an endogenous member of the mammalian family of RUNXs (RUNX1); this finding might indicate the possible pathogenesis of clonal hematopoiesis or myelodysplastic syndrome (MDS) upon marrow recovery [19]. There was no significant increase in MIP-1*α* after IST; this might have been due to the small sample size.

Eotaxin is also a CC chemokine and has been studied in bronchial asthma and many immune diseases [20]. An analysis of islet-infiltrating T cells in autoimmune diabetic syndrome demonstrated that the overexpression of pancreatic eotaxin, a typical Th2 chemokine, is associated with Th2-cell enrichment in insulitic lesions [9]. Of note, the RSAA patients experienced hyperfunction of the Th2 cytokines, which reversed their abnormally elevated Th1/Th2 ratios; eotaxin might play a similar role here. IL-1*β* and IL-1ra might play opposite roles and maintain the balance of the inflammatory response; therefore, the IL-1ra/IL-1*β* ratio is usually used in the study of other diseases such as coronary artery or central nervous system disease [21, 22]. In the present study, we found that IL-1ra levels and IL-1ra/IL-1*β* ratios were significantly higher in RSAA patients compared to HCs and SAA patients. Similarly, gene transfection of IL-1ra has been shown to inhibit degeneration and improve articular cartilage repair in osteoarthritis [23]. Recombinant human IL-1ra has also been observed to play a protective role in CCl4-induced acute liver injury in mice [24].

In correlation analysis, we observed that cytokine levels correlated with blood cell count in SAA and RSAA patients. Hemoglobin levels were only correlated with levels of MIP-1*α* and RANTES, possibly due to longer red blood cell life or erythrocyte transfusion in the early stage of SAA. Individual cytokines showed different correlation patterns with different blood cell types. In particular, IFN-*γ* and TNF-*α* negatively correlated only with absolute neutrophil count and platelet count, respectively. Meanwhile, PDGF-BB positively correlated only with platelet count; this result might indicate the source of cytokines and provide an experimental foundation for treatment aimed at a certain linage of SAA *in vivo*.

We performed analyses of the linkages between age/gender and cytokine concentrations, which revealed no significant differences in these linkages between SAA patients and healthy people. IL-8, IP-10, and FGF-*β* concentrations were associated with increasing age, and median IL-17 concentrations were higher for males than for females. There have been few reports on the relationships between these cytokines/chemokines and age/gender except in several age-related diseases, such as exudative age-related macular degeneration and age-related vocal fold atrophy [25, 26]. We have no specific explanation as to why the four cytokines and chemokines were related to age/gender. We also performed analyses of the linkages between age/gender and all of the 19 detected cytokines, and the results of these analyses were consistent with those of previous studies of healthy people [27, 28] (data not shown).

Measurements of cytokine concentrations before and after IST showed that eotaxin, IL-1ra, and MCP-1 concentrations increased earlier than MIP-1*β* and RANTES concentrations, and IFN-*γ* and G-CSF concentrations decreased earlier than IL-7, TNF-*α*, and IL-2 concentrations. The results of the correlation analysis of cytokine concentration with blood cells' count showed that IFN-*γ* and G-CSF significantly correlated with early recovery of absolute neutrophil count. Meanwhile, the absolute neutrophil count also recovered at the earlier time after IST in SAA patients in clinical practice. Corresponding phenomena were always observed in IL-2 and TNF-*α* concentrations, which significantly correlated with platelet count. In addition, cytokines with increased concentrations in the early stage after IST might play a stronger or more effective protective role in the immune pathogenesis of SAA than that in the later period and should be studied as a potential treatment strategy.

In summary, we examined the BMP concentrations of 27 cytokines using a Bio-Rad 27-Plex Luminex kit to evaluate the differences in the cytokine profiles of SAA patients and healthy people. The test results confirmed that Th1 cytokine levels were significantly increased and dominated in untreated SAA patients, while both Th1 and Th2 cytokine levels were increased. More importantly, we focused on cytokines and chemokines that were significantly elevated in RSAA patients and/or healthy people, such as MCP-1, IL-1ra, MIP-1, RANTES, PDGF-BB, and eotaxin. Future studies focusing on these cytokines and chemokines could help to create new, relevant laboratory examinations and provide a potential diagnostic or evaluation tool in clinical practice. Examinations that involve standard assays (e.g., ELISAs) to target these cytokines could be used more widely for the diagnosis and efficacy evaluation or prediction in SAA cases.

## Figures and Tables

**Figure 1:** Levels of cytokines and growth factors in the BMP of SAA patients, RSAA patients, and HCs. The bars represent median values. A rank-based Kruskal-Wallis one-way analysis of variance (ANOVA) was performed to test for differences in the concentrations of cytokines among SAA patients, RSAA patients, and HCs. SAA: severe aplastic anemia; RSAA: recovering SAA; HC: healthy control; ^*∗∗*^*p* < 0.01, ^*∗*^*p* < 0.05.

**Figure 2:** Different cytokine profiles of severe aplastic anemia (SAA) patients, recovering SAA (RSAA) patients, and healthy controls (HCs). A two-way hierarchical cluster analysis was performed on the log-transformed cytokine levels of SAA, RSAA, and HC samples using OriginPro 2018. Color scales represent cytokine levels (yellow indicates high levels; blue indicates low levels). The dendrogram above the figure was categorized into three clusters according to the cytokine profiles. The dendrogram to the left of the figure displays the proximities of the cytokines.

**Figure 3:** Correlation between cytokine concentration and age/gender. The 77 samples included samples from 36 males and 41 females, ranging in age from 11 to 78 years with a median age of 36 years.

**Figure 4:** Alternations of cytokine levels in SAA patients after immunosuppressive therapy (IST). In six SAA patients who responded to rabbit ATG + cyclosporine, BMP cytokine concentrations were measured before and three and six months after IST. Differences in cytokine levels before IST versus three months and six months after IST were assessed using an independent *t*-test or a Mann–Whitney *U* test depending on the data distribution ^*∗∗*^*p* < 0.01, ^*∗*^*p* < 0.05.

**Table 1:** Clinical and demographic parameters of patients participating in the present study.

Diagnosis	Number	Age (years)	ANC (10^9^/L)	Hb (g/L)	Plt(10^9^/L)	Ret%	Ret (10^9^/L)	Bone marrow karyotype	Therapy	Duration (months)
Untreated SAA	28	40 (11–78)	0.52 ± 0.82	74.39 ± 11.43	15.14 ± 10.44	0.68 ± 0.83	16.59 ± 19.89	Male 46, XY [9] Female 46, XX [9]	Not treated except for transfusions	2 (1–3)

Recovering SAA	19	26 (15–65)	4.65 ± 3.33	104.68 ± 37.32	77.42 ± 76.72	2.35 ± 1.16	68.42 ± 33.29	Male 46, XY [9] Female 46, XX [9]	Treated with a combination of ATG and CsA	32 (6–116)

Values are expressed as means ± SDs. Age and duration values are expressed as follows: mid (min–max). ANC: absolute neutrophil count; Hb: hemoglobin; Plt: platelet count; Ret: reticulocyte. Duration of untreated SAA: from the onset of disease to the time of cytokine measurement; duration of recovering SAA: from the onset of ATG therapy to the time of cytokine measurement.

**Table 2:** Statistical differences in the cytokine levels of SAA patients and HCs.

	SAA		RSAA		HC		*p* value
	Median	Mean ± SD	Median	Mean ± SD	Median	Mean ± SD	
IL-1*β*	0.25	0.60 ± 0.74	0.09	1.62 ± 6.04	0.40	1.19 ± 3.58	ns
IL-1ra	39.955	54.14 ± 50.87	120.72	190.63 ± 226.88	54.55	66.62 ± 54.05	0.002
IL-1ra/IL-1*β*	154.28	697.43 ± 1017.72	1211.00	6323.57 ± 10694.04	144.26	840.44 ± 1846.38	0.013
IL-2	1.69	2.85 ± 3.55	0.83	1.03 ± 1.02	0.605	0.63 ± 055	<0.001
IL-4	1.96	2.41 ± 1.85	2.31	2.46 ± 1.17	1.59	1.74 ± 0.63	ns
IL-7	20.17	19.99 ± 16.22	6.47	21.79 ± 47.52	10.22	15.65 ± 17.01	ns
IL-8	8.285	15.34 ± 13.80	11.46	79.21 ± 223.00	3.31	59.40 ± 182.72	ns
IL-9	10.53	19.17 ± 30.99	13.11	17.43 ± 18.61	18.69	21.50 ± 13.16	<0.001
IL-17	3.795	4.82 ± 3.26	6.84	7.15 ± 5.33	4.01	5.11 ± 2.58	ns
FGF-*β*	6.53	7.74 ± 4.83	5.94	7.06 ± 5.80	6.235	6.73 ± 2.61	ns
Eotaxin	52.125	64.78 ± 58.18	99.36	107.49 ± 80.50	53.415	59.07 ± 39.25	0.039
G-CSF	810.27	2518.84 ± 4163.51	84.32	191.90 ± 279.21	17.66	54.14 ± 94.76	<0.001
IFN-*γ*	3.56	5.19 ± 4.25	1.69	2.90 ± 3.12	1.51	1.84 ± 1.14	<0.001
IP-10	545.445	572.15 ± 356.15	442.08	460.00 ± 291.14	476.985	643.88 ± 515.86	ns
MCP-1	15.065	23.89 ± 23.02	9.47	18.36 ± 16.47	4.575	7.69 ± 8.39	<0.001
MIP-1*α*	2.635	3.96 ± 5.26	5.19	34.67 ± 104.49	2.31	27.57 ± 78.26	0.038
MIP-1*β*	26.895	32.58 ± 17.79	42.67	70.85 ± 79.20	46.32	76.94 ± 68.99	<0.001
PDGF-bb	96.85	236.80 ± 308.18	257.03	597.76 ± 1051.70	2492.395	2389.83 ± 1632.46	<0.001
RANTES	203.775	334.67 ± 366.43	1222.56	1299.58 ± 1162.78	1903.03	2027.68 ± 1201.01	<0.001
TNF-*α*	42.415	98.37 ± 178.04	27.96	28.16 ± 21.14	27.96	22.79 ± 17.69	0.003
IFN-*γ*/IL-4	1.89	2.50 ± 1.97	0.98	1.24 ± 0.84	0.885	1.13 ± 0.69	0.002

Data is presented in pg/ml; ns: not significant; SAA: severe aplastic anemia; RSAA: recovering SAA; HC: healthy control.

**Table 3:** Correlations of cytokines with blood cell counts in SAA and RSAA patients.

	ANC		Hb		Plt		Ret%		Ret	
IL-1ra	*r* = 0.613	*p* < 0.001	nc		*r* = 0.448	*p*=0.002	*r* = 0.323	*p*=0.027	*r* = 0.457	*p*=0.001
IL-2	*r* = −0.393	*p*=0.006	nc		*r* = −0.355	*p*=0.014	nc		*r* = −0.319	*p*=0.029
IL-9	nc		nc		*r* = 0.456	*p* < 0.001	*r* = 0.343	*p*=0.018	*r* = 0.302	*p*=0.039
IL-17	nc		nc		nc		nc		*r* = 0.290	*p*=0.048
Eotaxin	*r* = 0.381	*p*=0.008	nc		*r* = 0.348	*p*=0.017	*r* = 0.307	*p*=0.036	*r* = 0.355	*p*=0.014
G-CSF	*r* = −0.363	*p*=0.012	nc		*r* = −0.416	*p*=0.004	*r* = −0.521	*p* < 0.001	*r* = −0.498	*p* < 0.001
IFN-*γ*	*r* = −0.307	*p* < 0.001	nc		nc		nc		nc	
MIP-1*α*	*r* = 0.481	*p*=0.001	*r* = 0.389	*p*=0.007	*r* = 0.360	*p*=0.013	*r* = 0.510	*p* < 0.001	*r* = 0.595	*p* < 0.001
PDGF-bb	nc		nc		*r* = 0.480	*p*=0.001	nc		*r* = 0.338	*p*=0.020
MIP-1*β*	*r* = 0.442	*p*=0.002	nc		*r* = 0.424	*p*=0.003	*r* = 0.440	*p*=0.002	*r* = 0.500	*p* < 0.001
RANTES	*r* = 0.291	*p*=0.047	*r* = 0.414	*p*=0.004	*r* = 0.442	*p*=0.002	*r* = 0.451	*p*=0.001	*r* = 0.505	*p* < 0.001
TNF-*α*	nc		nc		*r* = −0.320	*p*=0.028	nc		nc	

ANC: absolute neutrophil count; Hb: hemoglobin; Plt: platelet count; Ret%: proportion of reticulocytes; Ret: absolute reticulocyte count; nc: no correlation.

## Data Availability

All the data used to support this study are available from the corresponding author upon request.
